The article "Medical Image Recognition Technology in the Effect of Substituting Soybean Meal for Fish Meal on the Diversity of Intestinal Microflora in Channa argus" was retracted in 2023. Reasons: signs of a paper mill; compromised peer review; unreliable results or conclusions.

# Medical Image Recognition Technology in the Effect of Substituting Soybean Meal for Fish Meal on the Diversity of Intestinal Microflora in *Channa argus*

**DOI:** 10.1155/2021/5269169

**Published:** 2021-11-25

**Authors:** Aixia Huang, Lihui Sun, Feng Lin, Jianlin Guo, Jianhu Jiang, Binqian Shen, Jianming Chen

**Affiliations:** Zhejiang Institute of Freshwater Fisheries, Huzhou, Zhejiang 313001, China

## Abstract

**Purpose:**

To study the application of medical image recognition technology based on backpropagation neural network (BPNN) in the effect of soybean meal replacing fish meal on intestinal microbial diversity of *Channa argus* and to evaluate the application value of this intelligent algorithm, *Channa argus* was fed with different contents of soybean meal instead of fish meal.

**Methods:**

After intestinal samples were collected and bacteria were isolated, microscopic imaging was performed, and the images were classified and identified. BPNN was constructed to perform denoising, smoothing, and segmentation.

**Results:**

After BPNN processing, the bacteria were completely separated from the original image background, and the bacteria was in the closed state, which was beneficial to feature extraction and species recognition. If there were 2 hidden layer nodes, the segmentation accuracy of bacterial microscopic images was the highest, up to 97.3%. With the replacement ratio of fish meal increased, the species of intestinal microbiome gradually enriched, and the relative abundance of intestinal microbiome was higher after fish meal was completely replaced by soybean meal (replacement). The intestinal microbial enzyme activities were affected by different fish meal and soybean meal contents in the diet. The glutamate transaminase and adenosine deaminase activities were increased after the replacement and were higher than those before the replacement, with statistically significant differences (*P* < 0.05).

**Conclusion:**

Replacement of fish meal with soybean meal has a significant effect on the intestinal flora diversity of *Channa argus*, and there is a close relationship between them. The image recognition technology based on BPNN has high recognition rate and segmentation accuracy for microbiological microscopic images.

## 1. Introduction

The colonization, establishment, composition, and diversity of intestinal flora are a complex process, which is a specific reflection of microorganisms in aquaculture water, feed, and environment [1]. Intestinal microbes have been proved to play an important role in regulating host immunity, metabolism, nutrient digestion, and absorption. Intestinal microbes of healthy fish can secrete a variety of digestive enzymes, such as protease, phosphatase, lipase, and cellulase, to help microbial hosts better absorb nutrients [2, 3]. As a host, fish inhabits a large number of microbial groups with characteristic functions. From the perspective of intestinal microorganisms, fish gut is its “fermenter,” and the undigested part of the food consumed by fish is its culture medium [4, 5]. In addition, fish gut microbes have the ability to encode genes that cannot be encoded by the host, and a wide variety of microbes in the fish gut plays a very important role in suppressing pathogenic microorganisms, which can protect the host fish from the invasion of pathogenic microorganisms [6, 7]. At present, the regulation of intestinal flora diversity of fish such as *Channa argus* has been gradually paid attention to. Related studies have found that adding probiotics to fish feed or water can significantly improve the performance, feed utilization rate, and immune ability of fish, adding lactobacillus with different treatment methods to the feed of *Channa argus*. Living lactic acid bacteria can better induce phagocytic activity and complement function of macrophages than heat-killing lactic acid bacteria and increase the level of plasma immunoglobulin [8, 9]. Fish meal with high protein content do not contain antinutritional factors, has good palatability, high digestibility, and amino acid balance, and contains many active factor, aquatic feedstuff industry in recent years [10]. However, it is not due to the fish powder production in China, and the fish powder resources are increasingly scarce and can meet the huge demand. Therefore, the fishery replacing fish powder is a more effective and correct strategy [11].

Image recognition technology is the one that processes and analyzes medical images using computer technology to identify and extract specific regions and targets [12]. The research goal is to classify the objects in the images based on the observed images and make judgments, that is, simulate the human cognition and understanding process using a computer [13, 14]. A general image recognition system is mainly composed of image segmentation, image feature extraction, and classifier recognition and classification [15]. With the help of image recognition technology, it can not only get information faster through image search but also produce a new way of interaction with the outside world and even make the outside world more intelligent operation [16]. Human vision has natural limitations. In some application scenarios, machine vision has advantages over human physiological vision, which is more accurate, objective, and stable [17, 18].

The computer intelligent image recognition technology is applied in the industrial detection or the recognition of medical images and biological microscopic images to realize the expansion of human visual function. In addition, the computer image recognition technology has the characteristics of high precision and accuracy and has high research significance and value. Therefore, in this study, it proposed a medical image recognition technology based on backpropagation (BP) neural network for the detection of intestinal flora diversity of Channa Argus, so as to study its application value.

## 2. Materials and Methods

### 2.1. Basic Data

*Channa argus* fishes were obtained from a commercial fish farm in Linghu town, China, and transported to our laboratory in Zhejiang Institute of Freshwater Fisheries, with a body weight of 95.71 ± 1.10 g. The fishes were reared in 15 cement ponds (3 m length × 2 m width × 1 m height) within recirculated freshwater with continuous aeration. The fish were fed with a commercial diet for 2 weeks to acclimate them to experimental conditions. The main protein sources of their diets were defatted fish meal and soybean meal. *Channa argus* fishes were randomly rolled into 5 groups: a group A (fish meal), a group B (soybean meal substituted 0.10 fish meal), a group C (soybean meal substituted 0.20 fish meal), a group D (soybean meal substituted 0.30 fish meal), and a group E (soybean meal substituted 0.40 fish meal), with 5 *Channa argus* in each group (Table 1). Each group of feeds was set with 3 replicates, and the experimental period was 84 d. Fishes were hand-fed to satiation twice daily (8 : 00 and 16 : 00). Water temperature ranged from 24 to 26°C during the feeding trial. In the feeding process, the residual food should be fished out in time to avoid affecting the water quality. At the end of the experimental, all the fishes were fasted for 24 hours and weighed.

### 2.2. Sample Collection

*Channa argus* fishes in each group were cleaned with medical alcohol and dissected in a sterile environment, and their intestines were taken out. The intestines were tied tightly with sterile fine thread on both sides, and the outer wall of the intestines was wiped with 75% alcohol cotton and then rinsed for several times. Then, the intestines of *Channa argus* were cut open; the contents were gently squeezed out and then rinsed with sterile water again. The intestinal contents and intestinal mucosa samples of each group were mixed and preserved in liquid nitrogen.

The intestinal microflora of *Channa argus* were detected by adding 1 mL phosphate buffer (PBS) and 20 *μ*L 20% polyvinylpyrrolidone (PVPP) homogenate. Centrifugation was carried out at 200 RPM for 6 min, supernatant was taken, and 1 mL PBS was added to the lower layer of precipitation; supernatant was taken after centrifugation again, and supernatant was combined with supernatant solution and centrifuged at 300 RPM for 6 min; supernatant was taken and centrifuged at 1200 RPM for 6 min; then, bacteria was collected and washed with PBS. 300 *μ*L lysate I, 10% lysozyme 100 *μ*L, and 1% RNA nuclease (RNase) 20 *μ*L were added to the obtained cell after washing, and the mixture was kept for half an hour at 37°C. 300 *μ*L cracking solution II, 50 *μ*L20% sodium dodecyl sulfate (SDS), and 50 *μ*L20%PVPP were added, mixed, and kept in ice bath for 5 min. Equal volume of phenol/chloroform was added and centrifuged at 13000 RPM for 8 min; then, the supernatant was taken, operation was repeated once again; 2 times the volume of isopropyl alcohol and 1/10 of 3M sodium acetate were added and precipitated for 2 h at −20°C. Centrifugation was performed at 14000 RPM at 4°C for 10 min, and supernatant was removed and dried under a super clean platform, resuspended, and frozen at −80°C.

The PCR primer was a nearly full-length universal bacterial primer: 27F (5′-AGAGTTTGATCMTGGCTC-3′; M = A or C) and 13878 (5′- GGGCGGWGTGTACAAGGC - 3′; W = A or T). The extracted genomic DNA was diluted 20 times to take 1, 2, 4, and 8 *μ*L and the original sample was 1 *μ*L and 2 *μ*L as templates, respectively. The PCR reaction system was as follows: sterile double distilled water 34.5 *μ*L, 10 × PCR buffer 5 *μ*L, 2.5 mmol/L dNTP 4 *μ*L, 2.5 *μ*mol/L PCR primers 2 *μ*L each, and Taq enzyme 0.5 *μ*L. Reaction conditions: pre-denaturation at 94°C for 4 min, 94°C for 1 min, 55°C for 1 min, 72°C for 2 min, 30 cycles, and 72°C for 10 min. 5 *μ*L PCR amplification products were selected for 1.2% agarose gel electrophoresis, DNA Marker DL2000, UV detection amplification products, and gel imaging. Finally, Project Classifier V.2.2 was used to perform cluster analysis (genus and species of microorganisms) on the representative sequences.

### 2.3. Preprocessing of Bacterial Microscopic Images

The algebraic operation before image segmentation is aimed at adding, subtracting, multiplying, and dividing the obtained image through point-to-point method and the image is output. The operation method is shown in equations (1)–(4):

(1) $$\begin{array}{c} T\left(a,b\right)=I_{1}\left(a,b\right)+I_{2}\left(a,b\right), \end{array}$$

(2) $$\begin{array}{c} T\left(a,b\right)=I_{1}\left(a,b\right)-I_{2}\left(a,b\right), \end{array}$$

(3) $$\begin{array}{c} T\left(a,b\right)=I_{1}\left(a,b\right)\times I_{2}\left(a,b\right), \end{array}$$

(4) $$\begin{array}{c} T\left(a,b\right)=\frac{I_{1}\left(a,b\right)}{I_{2}\left(a,b\right)}, \end{array}$$

where *I*_1_(*a*, *b*) and *I*_2_(*a*, *b*), respectively, represent two input images to be operated on and *T*(*a*, *b*) is the output image. In order to complete the noise reduction of the output image, noise reduction can be achieved by adding and canceling the noise objects for many times [19]. If the microscopic image is composed of *N* images, its image form is as follows:

(5) $$\begin{array}{c} P_{i}\left(a,b\right)=Q\left(a,b\right)+Z_{i}\left(a,b\right), \end{array}$$

where *Q*(*a*, *b*) is an ideal denoised image and *Z*_*i*_(*a*, *b*) is the image before denoising. It is assumed that all *n* images come from the same sample set of random noise images with a noise mean of 0, namely,

(6) $$\begin{array}{c} \varepsilon \left\{Z_{i}\right.\left.\left(a,b\right)\right\}=0. \end{array}$$

Power signal noise is shown in equation (7):

(7) $$\begin{array}{c} W\left(a,b\right)=\frac{S^{2}\left(a,b\right)}{\varepsilon \left\{Z^{2}\right.\left.\left(a,b\right)\right\}}. \end{array}$$

If the above *n* images are averaged (as shown in equation (8)), the average SNR is shown in equations (9) and (10):

(8) $$\begin{array}{c} \bar{X}\left(a,b\right)=\frac{1}{n}\sum_{i=1}^{n}\left[Q\left(a,b\right)+Z_{i}\left(a,b\right)\right], \end{array}$$

(9) $$\begin{array}{c} \bar{W}\left(a,b\right)=\frac{S^{2}\left(a,b\right)}{\varepsilon \left\{\left(1/n\right)\sum_{i=1}^{n}{\left[Z_{i}\left(a,b\right)\right]}^{2}\right\}}, \end{array}$$

(10) $$\begin{array}{c} \bar{W}\left(a,b\right)=\frac{n^{2}S^{2}\left(a,b\right)}{n\varepsilon \left\{Z^{2}\left(a,b\right)\right\}}=nW\left(a,b\right). \end{array}$$

The average signal-to-noise ratio of each point in the image is increased *n* times by averaging *n* images.

### 2.4. Bacterial Identification Based on BPNN

BPNN covers an input layer, a hidden layer, and an output layer, as shown in Figure 1. The neurons in each layer are fully connected with those in the adjacent layer, and there is no feedback connection among them, thus forming a feedforward neural network system with hierarchical structure.

In the BPNN, the input layer contains a node and the output layer contains B nodes, so it can be regarded as a mapping from a dimension vector to *a* dimension vector *b*. The number of nodes in the hidden layer can be calculated as follows:

(11) $$\begin{array}{c} N=\sqrt{a+b}+C, \end{array}$$

where *n, a,* and *b* refer to the number of nodes in hidden, input, and output layer, respectively, and *c* represents the adjustment constant. The relationship between output and input of the BPNN is given as follows:

(12) $$\begin{array}{c} {\text{net}}_{u}=\sum_{v=1}^{b}Q_{uv}I_{v}-p,\\ O_{u}=A\left({\text{net}}_{u}\right), \end{array}$$

where *I* represents the input signal transmitted by neurons, *Q* represents the connection weight between neurons, *P* represents the offset, *O* represents the output of neurons, *A* is the activation function, and then net is the net activation. It is supposed that there is a neural network in layer *a* and sample *m* is added at the input layer. The sum of inputs of *u* neurons in layer *n* is *S*_*u*_^*n*^ and the output is *I*_*u*_^*n*^. The weight coefficient of the *v* neuron in layer *n* − 1 to the *u* neuron in layer NTH is *Q*_*uv*_, and the firing function of each neuron is *A*:

(13) $$\begin{array}{c} A\left(m\right)=\frac{1}{1+\exp\left(-m\right)}. \end{array}$$

Relationship between variables can be expressed mathematically as follows:

(14) $$\begin{array}{c} m_{u}^{n}=A\left(S_{u}^{n}\right),\\ S_{u}^{n}=\sum_{v}Q_{uv}m_{v}^{n-1}. \end{array}$$

It points toward the BPNN algorithm, and backpropagation travels two steps forward according to the order in which each layer is spread; the actual output and desired output are compared; if there is a difference in backpropagation, the weight coefficient of each neuron in the hidden layer is modified according to the propagation of the positive path to minimize the error signal, and the weight coefficient of each neuron in hidden layer is modified. The error signal is minimized.

BP error function is defined as equation (15), and its gradient is determined to be (16):

(15) $$\begin{array}{c} r=\frac{1}{2}{\sum_{u}\left(I_{u}^{a}-O_{u}\right)}^{2},\\ \frac{\partial r}{\partial Q_{uv}}=\frac{\partial r}{\partial S_{u}^{n}}\cdot \frac{\partial S_{u}^{n}}{\partial Q_{uv}}, \end{array}$$

(16) $$\begin{array}{c} r=\frac{1}{2}{\sum_{u}\left(I_{u}^{a}-O_{u}\right)}^{2},\\ \frac{\partial r}{\partial Q_{uv}}=\frac{\partial r}{\partial S_{u}^{n}}\cdot \frac{\partial S_{u}^{n}}{\partial Q_{uv}}, \end{array}$$

where ∂*S*_*u*_^*n*^/∂*Q*_*uv*_=*I*_*v*_^*n*−1^, *r* refers to the error of backpropagation, *Q* refers to the weight, and *Ou* is the output of neuron *U*; let *d*_*u*_^*n*^=∂*r*/∂*S*_*u*_^*n*^; then,

(17) $$\begin{array}{c} \frac{\partial r}{\partial S_{u}^{n}}=\frac{\partial r}{\partial I_{u}^{n}}\cdot \frac{\partial I_{u}^{n}}{\partial S_{u}^{n}}, \end{array}$$

where *Iu* refers to the input of neuron *u*, *S*_*u*_^*n*^ represents sum of input of neuron *u* in layer *n*, ∂*I*_*u*_^*n*^/∂*S*_*u*_^*n*^=*A*′(*S*_*u*_^*n*^), *A*′(*S*_*u*_^*n*^)=(1/1+exp(−*S*_*u*_^*n*^))′, and (1/1+exp(−*S*_*u*_^*n*^))′=*I*_*u*_^*n*^(1 − *I*_*u*_^*n*^). When *n* = *a* in the equation, ∂*r*/∂*I*_*u*_^*n*^=∂*r*/∂*I*_*u*_^*a*^. When *n* < *a*, ∂*r*/∂*I*_*u*_^*n*^=∑_1_∂*r*/∂*S*_1_^*n*+1^ · ∂*S*_1_^*n*+1^/∂*I*_*u*_^*a*^ and ∑_1_∂*r*/∂*S*_1_^*n*+1^ · ∂*S*_1_^*n*+1^/∂*I*_*u*_^*a*^=∑_1_*Q*_*Iu*_ · *d*_1_^*n*+1^.

Therefore, the modified equation of the weight of the neural network is

(18) $$\begin{array}{c} \Delta Q_{uv}\left(t+1\right)=\alpha \Delta Q_{uv}\left(t\right)-\theta \cdot d_{1}^{n}\cdot I_{v}^{n-1}. \end{array}$$

If *I*_*u*_^*n*^=*e*, then *d*_1_^*n*^=*I*_*u*_^*n*^(1 − *I*_*u*_^*n*^)∑*Q*_*Iu*_*·d*_1_^*n*+1^, where *Q* is the weight, *I* refers to the input, *r* is the propagation error, and *a* is the number of nodes in the input layer.  Figure 2 is the schematic diagram of the algorithm to segment the bacterial fiber image.

### 2.5. Effect Evaluation

In this study, the BPNN algorithm was experimentally verified and used for abdominal MRI image segmentation of patients with intestinal obstruction. Based on the segmentation technology of graph cutting, the image was mapped into a network image, and the segmentation problem was transformed into different operations on the image. The maximum flow/minimum cutting theorem was used to realize the segmentation of the image. In addition, the edge detection algorithm and threshold segmentation algorithm are introduced, and the application value of BPNN in MRI image segmentation of intestinal obstruction is analyzed through comparison.

### 2.6. Statistical Method

SPSS 22.0 was selected for data processing. The measurement data were expressed in the form of mean ± standard deviation ($\overset{–}{x}$ ± *s*), and the counting data were displayed as percentage (%). One-way ANOVA was used to analyze the data difference between groups, and *P* < 0.05 meant that the difference was statistically significant.

## 3. Results

### 3.1. Common Bacteria in the Intestine of *Channa argus*

Figure 3 shows several common bacteria in the intestinal flora of *Channa argus*. The intestinal flora includes symbiotic bacteria (probiotics, which assist the gastrointestinal tract in metabolism, decomposition, digestion, and absorption), opportunistic pathogens (between symbiotic bacteria and pathogenic bacteria), and pathogenic bacteria (which directly cause digestive tract diseases). Figure 3 below shows the electron microscopic morphology of symbiotic bacteria, opportunistic pathogens, and pathogenic bacteria.

### 3.2. Segmentation of Microscopic Images of Bacteria

The bacteria images extracted from the system are preprocessed and gray-level equalized by BPNN and then segmented.  Figure 4 shows the bacteria images after a different processing. It can be seen that the background of the bacteria after segmentation by BPNN is completely separated from the original image, and the bacteria are in a closed state, which is beneficial to its feature extraction and species recognition.

### 3.3. Segmentation Effect of the Image

In BPNN, the number of nodes in the hidden layer can determine the effect of image segmentation to a certain extent.  Table 2 shows the image segmentation accuracy of BPNN with different hidden layer nodes. The segmentation accuracy of bacterial microscopic images is the highest, reaching 97.3% when there are 2 nodes in the hidden layer.

### 3.4. Analysis of Intestinal Microbial Diversity of *Channa argus*

The five groups of *Channa argus* were fed with 0%, 10%, 20%, 30%, and 40% soybean meal instead of fish meal for 3 weeks, respectively. The intestinal samples of *Channa argus* were collected, and the microbial diversity of the intestinal flora was analyzed. The results in Figure 5 illustrated that, with the increase of the replacement ratio of fish meal, the species of intestinal microflora were gradually enriched, and the relative abundance of intestinal microflora was higher after fish meal was completely replaced by soybean meal.

### 3.5. Change of Intestinal Microbial Enzyme Activity

Figure 6 shows the grain third transaminase and adenosine deaminase activities were different in the feed gut microbial soybean meal; the changes in different fish meal and soybean meal content affected the intestinal microbial enzyme activity. Both the grain third transaminase meal promotion and adenosine deaminase activity after soybean meal replacement (group E) were higher than the one before (group A) (*P* < 0.05).

## 4. Discussion

Healthy gastrointestinal tract is very important for overall health, and animal health depends on the intake of nutrients, the balance of digestive juice (acid and enzyme), and the important role of microorganisms in the digestive system [20]. The research on promoting microecology in aquatic animals is still in its infancy, but its importance has been recognized and related research has been carried out [21, 22]. Facing the current situation of rapid development and large scale of China's animal husbandry and feed industry, in order to reduce the dependence of China's feed industry on fish meal and other expensive animal protein sources, it is very important to develop cheaper and easily available protein products to meet the animal's needs for feed protein nutrition [23, 24]. Soybean meal is an important vegetable protein source because of its rich nutrients. The soybean protein content in soybean meal is between 43.0% and 55.0%, and most of them are water-soluble proteins. Besides protein, they also contain other rich nutrients, which is a good dietary protein source for fish and monogastric animals [25, 26]. Therefore, it is of crucially practical significance to explore the effects of soybean meal instead of fish meal on the intestinal microbial diversity of fish.

In this study, after *Channa argus* was fed with soybean meal instead of fish meal, its intestinal samples were collected and bacteria were separated, and then microscopic images were classified and identified. By constructing BPNN, various kinds of dryness removal and smoothing processing were carried out on the images according to various noises existing in the microscopic images and the requirements of image color normalization. The change of intestinal flora diversity of *Channa argus* was analyzed by image segmentation and recognition. As a result, the background of the segmented bacteria is completely separated from the original image, and the bacteria are in a closed state, which is beneficial to feature extraction and species recognition. When 2 nodes are set in the hidden layer, the segmentation accuracy of the bacteria microscopic image is the highest, reaching 97.3%. That is to say, the image recognition technology based on BPNN has high recognition and segmentation performance for bacterial microscopic images, and the segmentation effect is good, which is beneficial to the recognition of microbial species and diversity analysis. Different contents of fish meal and soybean meal in the feed affected the intestinal microbial enzyme activity. After replacing fish meal with soybean meal (Group E), the activities of alanine aminotransferase and adenosine deaminase increased and were higher in contrast to those before replacement (Group A) (*P* < 0.05). The results of Rimoldi et al. [27] are similar to those of. The results show that the microbial fermentation of soybean meal instead of fish meal not only improves the activities of glutamic-pyruvic transaminase and adenosine deaminase in the intestinal tract of *Channa argus* but also has a great influence on the intestinal microbial diversity, that is, there is a close relationship between the protein content in the feed and the intestinal flora diversity.

## 5. Conclusion

The results of this study show that soybean meal instead of fish meal had a great influence on the diversity of intestinal flora of *Channa argus*, and there was a close relationship between them. Image recognition technology based on BPNN had high recognition rate and segmentation accuracy for microbial microscopic images. In a word, this study provides a reference for the application of intelligent algorithms such as BPNN in the effect of replacing fish meal with soybean meal on the intestinal microbial diversity of *Channa argus*.

## Figures and Tables

**Figure 1:** Recognition process of the bacterial microscopic image.

**Figure 2:** Preprocessing of fiber image. (a) The original picture taken. (b) Pretreatment. (c) Bacterial image after feature extraction and segmentation.

**Figure 3:** Common bacteria in the intestine of *Channa argus*. (a), (b), and (c) Bacteroides, lactobacillus, and bifidobacterium, respectively; (d), (e) and (f) Staphylococcus, *Escherichia coli*, and streptococcus, respectively. (g) and (h) Salmonella and *Helicobacter pylori*, respectively.

**Figure 4:** Segmentation of microscopic images of bacteria. (a) Micrograph of bacteria extracted by the system. (b) The image after grayscale equalization. (c) The segmented image.

**Figure 5:** Common bacteria in the intestine of *Channa argus*. A, B, C, D, and E refer to different groups. a∼k represent Acinetobacter, Bacillus, Carnobacterium, Clostridium, Geobacillus, Pseudomonas, Leuconostoc, Thermomonas, Planctomyces, Streptococcus, and other genera, respectively.

**Figure 6:** Activities of glutamic-pyruvic transaminase and adenosine deaminase in intestinal microorganisms of *Channa argus*. *Note*. ^*∗*^means significant difference compared with A group (*P* < 0.05).

**Table 1:** Protein source of *Channa argus* feed.

Group	Fish meal (%)	Soybean meal (%)
A	100	0
B	90	10
C	80	20
D	70	30
E	60	40

**Table 2:** Accuracy of image segmentation.

Number of nodes	Accuracy (%)
2	97.3
3	96.5
4	94.8
5	94.8
6	94.8
7	94.1
8	94.1

## Data Availability

The data underlying the results presented in the study are available within the article.
